RETRACTED

# Antitumor Proliferation and Related Mechanism of Ultrasound Irradiation Combined with Safflower Yellow

**DOI:** 10.1155/2022/5168886

**Published:** 2022-06-16

**Authors:** Gen Li, Lijun Xu, Xiaoli Wang

**Affiliations:** ^1^Division of Cardiothroracic and Vascular Surgery, Tongji Hospital, Tongji Medical College, Huazhong University of Science and Technology, Wuhan 430030, Hubei, China; ^2^Cancer Biology Research Center, Tongji Hospital, Tongji Medical College, Huazhong University of Science and Technology, Wuhan 430030, Hubei, China; ^3^Department of Obstetrics and Gynecology, Tongji Hospital, Tongji Medical College, Huazhong University of Science and Technology, Wuhan 430030, Hubei, China

## Abstract

Ultrasound irradiation is now the best method for evaluating benign and malignant tumor nodules. Chemotherapy has always played an important role in the treatment of malignant tumors. With the large-scale application of chemotherapy drugs, the problem of multidrug resistance of tumors has become more and more prominent, which has become one of the difficulties in tumor chemotherapy. This study mainly explores the antitumor proliferation and related mechanisms of ultrasound irradiation combined with safflower yellow. The breast cancer cell line 4T1 derived from BALB/c mice was selected. BALB/c is an albino laboratory mouse, which, like many commonly used sublines, originated from Mus musculus. BALB/c mice have been bred for more than 200 generations in research institutions around the world and are widely used in animal experiments in immunology and physiology. When the cell proliferation reached 80%–90% of the bottom area of the culture flask, it was resuspended, passaged, frozen, and resuscitated according to experimental needs. The 4T1 breast cancer cell line was cultured by conventional methods. 4T1 breast cancer cells in the logarithmic proliferation phase were collected. After 0.25% was digested with pancreatin, it was washed twice with PBS to adjust the concentration to 1 × 10^7^/mL. A 0.1 mL tumor cell suspension was subcutaneously inoculated on the edge of the mouse chest, thereby establishing a breast cancer model of BALB/c mice. After 6-15 days, the tumor volume grew rapidly and became larger. When the length of the tumor is 2.5 × 2.5, the modeling is successful. Ultrasound-targeted microbubble destruction technology, as a novel drug delivery method with high efficiency and low toxicity, can form transient pores (sonoporation effect) on the cell surface, widen the intercellular space, and increase the membrane permeability, and thus effectively. The transport of drugs, genes, proteins, etc., is promoted to target organs and tissues. Tumor-forming mice were randomly divided into the following four groups: control group, safflower yellow group, ultrasound irradiation group, and ultrasound irradiation combined with safflower yellow group. From the second day of inoculation to the end of the experiment, the body weight of the mice successfully inoculated with 4T1 cells was measured every day; from the 5th day, tumors in each group were calculated body volume and tumor inhibition rate (TIR) of each group. The combined treatment group has a higher tumor inhibition rate than the ultrasound irradiation group, and the difference is statistically significant (*P* < 0.05). Ultrasound irradiation combined with safflower yellow pigment can effectively inhibit tumor proliferation, maintain, or even improve the efficacy of chemotherapy, thereby improving the patient's tolerance to chemotherapy.

RETRACTED

## 1. Introduction

Breast tumors show different pathological signs according to the type of tissue. Compared with ordinary cells, tumor cells have higher ultrasound sensitivity and are better targets for drug-targeted therapy mediated by ultrasound. Using the “sonic pore effect” of microbubble blasting can increase the permeability of local microvessels and cell membranes, promote the penetration of drugs, and then increase the accumulation of chemotherapeutic drugs in target tissues. The intracellular concentration of chemotherapeutic drugs increases the cytotoxicity of chemotherapeutic drugs.

In some studies, the location of the tumor is also a predictor of benign and malignant breast lesions. Chemotherapy has always occupied an important position in the treatment of malignant tumors. With the large-scale application of chemotherapy drugs, the problem of multidrug resistance of tumors has become more and more prominent, which has become one of the difficulties in tumor chemotherapy. Tumor multidrug resistance often occurs when tumor patients receive chemotherapy, which is induced by a certain drug, and exhibits cross-resistance to other anticancer drugs with completely different structures and mechanisms.

There is an urgent need to develop new drugs to overcome this drug resistance, improve the therapeutic effect, and reduce the side effects caused by the treatment of tumors. In recent years, traditional Chinese medicine has been proven to have great potential in tumor treatment and has received more and more attention. In recent years, the treatment of tumors has always been a concern of people. O'Shea et al. introduced the basic technology of motion estimation in the United States and its current clinical applications in the prostate, as well as the latest technology. He integrates these technologies into the functions of the RT workflow easily, at low cost and effectively. Although his research imaging technology can ultimately contribute to many, the research process lacks data to support [1]. Lichtenstein believes the equipment to continuously measure flow and trigger a new echocardiographic evaluation. Although he should perform echocardiography, the study did not give out the factors affecting diastolic function [2]. The research of Meng et al. is only reflected in male patients, so the research process is relatively one-sided [3]. Huang et al. proposed a novel ultrasound image segmentation variation mode, and there is no experimental control in the research process [4]. Chemotherapy is one of the traditional methods for the treatment of tumors, but the efficacy of chemotherapy is limited, and chemotherapy drugs are prone to drug resistance, have serious adverse reactions, and will continue to affect the therapeutic effect of chemotherapy drugs [5, 6].

RETRACTED

The breast cancer cell line 4T1 derived from BALB/c mice was selected. When the cell proliferation reached 80%–90% of the bottom area of the culture flask, it was resuspended, passaged, frozen, and resuscitated according to experimental needs. The 4T1 breast cancer cell line was cultured by conventional methods. The content of the innovation point is not very complete, and I have added some content. After inoculation with transplanted tumor cells for a period of time, all mice were sacrificed and routinely sterilized, and the subcutaneous tumors in the left flank of the mice were completely excised [7, 8]. 4T1 breast cancer cells in the logarithmic proliferation phase were collected. After 0.25% was digested with pancreatin, it was washed twice with PBS to adjust the concentration to 1 × 107/mL. A 0.1 mL tumor cell suspension was subcutaneously inoculated on the edge of the mouse chest, thereby establishing a breast cancer model of BALB/c mice. After 6–15 days, the tumor volume grew rapidly and became larger. When the length of the tumor is 2.5 × 2.5, the modeling is successful. From the second day of inoculation to the end of the experiment, the body weight of the mice successfully inoculated with 4T1 cells was measured every day; from the 5th day, tumors in each group were calculated body volume and tumor inhibition rate (TIR) of each group.

## 2. Antitumor Proliferation

### 2.1. Ultrasound Irradiation

As a noninvasive treatment technology emerged in recent years has been widely used at home and abroad and has achieved significant clinical effects, EUS is also used in tumor staging to guide treatment decisions for patients with esophageal cancer. In CEUS, the TIC curve comprehensively reflects the amount of contrast agent in the diseased area, the invasion speed, and the internal microcirculation of the tumor. The relevant influencing factors *α* of the TIC curve are expressed as follows [9, 10]:

(1) $$\begin{array}{c} \alpha =\frac{\text{log}\left(B_{m}/B_{n}\right)-\delta }{2\left(n-m\right)x}\left(\text{db}/\text{mm}\right)\left(n=0,1,2\ldots k\right), \end{array}$$

where *B*_*m*_ is the number of contrast agents. For malignant tumors, as the volume of the tumor increases, the full length of the angiogenic part will double, and the internal pressure of the tumor will double, which is connected to the tumor's rich blood supply. Cancer can easily become an aneurysm due to its abundant new blood vessels, weak tube wall and lack of muscle layer, disordered vascular branches, and irregular lumens. Therefore, the contrast image of cancer lesions before chemotherapy shows ultrahigh intensity and rapid inflow of contrast agent and flow of arteries. After using contrast agent chemotherapy, the residual lesions showed degenerative changes, the cancer cells became fewer, the interstitium often became fibrous, the mucus was degenerated or showed glass-like changes, the appearance of new blood vessels, the decrease in vascular elasticity, and the end of vascular occlusion, and the above diseases physiological changes lead to the insufficient blood supply and result in residual disease. The use of ultrasound contrast can indicate changes in blood flow velocity and number of blood vessels [11].

(2) $$\begin{array}{c} P=\frac{p_{0}F_{s}}{2\lambda x}\sqrt{\frac{D_{s}}{2x}}+\frac{4Z_{1}Z_{2}}{{\left(Z_{2}+Z_{1}\right)}^{2}}\left(X_{m}-X_{n}\right), \end{array}$$

where *p*_0_ is the initial contrast. The propagation process of ultrasound needs to follow the corresponding propagation law [12, 13].

(3) $$\begin{array}{c} \frac{\sin\;\alpha_{L}}{c_{L1}}=\frac{\sin\;\alpha^{m}{}_{L}}{c_{L1}}\\ =\frac{\sin\;\alpha_{s}}{c_{L1}}=\frac{\sin\;\beta_{L}}{c_{s2}}=\frac{\sin\;\beta_{s}}{c_{s1}}, \end{array}$$

where *β* is the corresponding angle, and *c* is the angle coefficient. Traditional ultrasound can only see the morphological changes of cancer lesions, and it is difficult to accurately evaluate the internal functional changes caused by chemotherapy drugs such as the reduction of blood vessels, the formation of nonliquefied necrotic areas, and the formation of fibrous lesions. However, this change is often an effective sign of early chemotherapy. Contrast-formed ultrasound is used as an imaging method for blood characteristics [14, 15]. The incidence of allergies is low, and the discharge is fast during breathing. It has the characteristics of reducing the excretion burden of the liver and kidneys. The characteristics of the internal medium can clearly indicate that it is a tumor blood vessel, which can be clearly displayed after chemotherapy. The quality and quantity of blood inside the tumor are very useful for the treatment of cancer, and it may become the main way to treat NAC. In tumor elastography, on the one hand, due to hardness testing and noninvasive treatment methods, simple operations and experiments can be repeated to reduce the rate of malignant tumors, making benign and malignant tumors after cancer treatment an auxiliary diagnosis of NAC. Very high heat is generated during tumor proliferation [16].

(4) $$\begin{array}{c} J=-\frac{1}{m}\left[\sum_{i=1}^{m}\sum_{k=1}^{K}y_{k}\text{log}\left(h_{0}\left(x\right)\right)+\left(1-y_{k}\right)\text{log}\left(1-\left(h_{0}\left(x\right)\right)\right)\right], \end{array}$$

where *J* is the heat generated during tumor proliferation. If wwww, then the loop is terminated, and there are [17, 18]

(5) $$\begin{array}{c} M\left(x\right)=\sum_{t=1}^{T}\beta^{t}h^{t}\left(x\right). \end{array}$$

Tumor calcification means that the tumor morphology has changed. Many studies believe that the larger the calcified particles, the better the differentiation of the cancer tissue. and the lower the degree of malignancy [19, 20]. During the treatment process, the tumor, necrotic area, fibrosis area, and hardness may undergo subtle changes. Since it is invisible to the naked eye, NAC elastography has become one of the adjuvant treatment methods for cancer. In the early stage of cancer, because there are no small nodules, the lesions are all appearing in hidden places, and there are no obvious clinical symptoms, so it is difficult to find. According to high-frequency ultrasound technology, the detection rate of tumor nodules has increased. Most studies have shown that the suspected malignant symptoms of tumor nodules under ultrasound mainly include microcalcification, hypoechoic, solid nodules, irregular shapes, uneven or fuzzy boundaries, and intracellular diffusion [21]. The ultrasonic irradiation equipment is shown in Figure 1.

RETRACTED

*N* independent individual neural networks:

(6) $$\begin{array}{c} Q_{err}=\sum_{k>1/2}C_{N}^{k}p^{k}{\left(1-p\right)}^{k}. \end{array}$$

The larger the *N*, the smaller the *Q*_*err*_ [22, 23]:

(7) $$\begin{array}{c} w_{i}=\frac{1}{M}. \end{array}$$

Calculate *h*^(*t*)^ [24, 25]:

(8) $$\begin{array}{c} e^{\left(t\right)}=\sum_{t=1}^{m}w^{\left(t\right)}\left|y_{t}-h^{\left(t\right)}\left(x_{i}\right)\right|,\\ \beta^{\left(t\right)}=\frac{e^{t}}{1-e^{t}},\\ w_{i}^{\left(t+1\right)}=w_{i}^{\left(t\right)}{\left(\beta^{\left(t\right)}\right)}^{1-\left|y_{i}-h_{i}^{\left(t\right)}\left(x_{i}\right)\right|}. \end{array}$$

### 2.2. Carthamus Yellow

Safflower (Crcrthr11s linctoriusL) is a traditional Chinese medicine used to treat cardiovascular disease, stroke, and angina pectoris [26, 27]. Hydroxysafflor yellow A is one of the main active ingredients of safflower. It has been reported that it is a blood circulation disorder. There are studies that have proved that hydroxysafflor yellow A is effective for liver cancer, glioma, and colorectal cancer. A variety of tumor cells have therapeutic effects, but there is no report on clinical tumor research [28]. So far, more than 200 compounds have been isolated and identified from safflower, among which flavonoids are the main components of the above-mentioned therapeutic effects [29, 30]. Recently, a new quinolone c-glycoside was isolated from safflower, called hydroxysafflor yellow B (HSYB), which is an isomer of hydroxysafflor yellow A. Phytochemical and pharmacological studies have shown that HSYB has antioxidant effects [31]. Traditional Chinese medicine believes that tumors are caused by the imbalance of qi and blood in the human body, causing pathological changes such as qi stagnation and blood stasis [32, 33]. Tumors refer to new organisms formed by the proliferation of local tissue cells under the action of various tumorigenic factors because these new organisms are mostly space-occupying massive protrusions, also known as neoplasms.

Let *T*=*t* − 1 [34]

(9) $$\begin{array}{c} H\left(x\right)=\text{sign}\left(\sum_{i=1}^{t}\beta^{\left(t\right)}h^{\left(t\right)}\right). \end{array}$$

Enter *M* data samples with category labels, and let

(10) $$\begin{array}{c} D=\left\{\left(x_{1},y_{1}\right),\ldots \left(x_{M},y_{M}\right)\right\}. \end{array}$$

Estimate the efficacy of *h*^(*t*)^:

(11) $$\begin{array}{c} e^{\left(t\right)}=\sum_{t=1}^{M}w_{i}^{\left(t\right)}\left|y_{i}-h_{i}^{\left(t\right)}\left(x_{i}\right)\right|,\\ w_{i}^{\left(t+1\right)}=\frac{w_{i}^{\left(t\right)}\text{exp}\left\{-\beta^{\left(t\right)}y_{i}h_{i}^{t}\left(x_{i}\right)\right\}}{Z_{t}}. \end{array}$$

Among them, the activation value is

(12) $$\begin{array}{c} y=\frac{2}{\left[1-\text{exp}\left(-2x\right)\right]-1}. \end{array}$$

## 3. Antitumor Proliferation and Related Mechanism Experiments

### 3.1. Selection and Cultivation of Cell Lines

#### 3.1.1. Selection of Cell Lines

The name of breast cancer cell line 4T1 is derived from BALB/c mice. In addition, the mice were reared adaptively for 1 week and kept in a clean cabinet with free drinking water and food. All mouse experiment operations strictly follow the laboratory animal management regulations.

RETRACTED

Preparation of hydroxysafflor yellow B mother liquor: use a precision electronic balance to accurately weigh 20 mg of hydroxysafflor yellow B powder and place it in a 1.5 mL EP tube, use a pipette to extract 200 *μ*L of DMSO solution and the HSYB powder in the EP tube to fully dissolve it, formulated it into a 100 mg/mL experimental mother liquor, and during the dissolution period, use a vortexer at 500 rpm, 10 s to help the two to fully blend.

Preparation of DMEM complete medium: add 50 mL of normal fetal bovine serum to 445 mL of HyClone basic medium and use a pipette to gently rotate and mix during the process of adding serum. After the two are completely mixed, add 1%, that is, 5 mL penicillin-streptomycin mixing solution (100x), and after the three are completely blown, it is made into a 500 mL DMEM complete medium. Use sterile 50 mL centrifuge tubes to pack the complete medium for normal use and prevent contamination. The centrifuge tube and the remaining medium are stored in a 4°C refrigerator and protected from light and low temperature.

The preparation of phosphate buffer saline (PBS): use a precision balance to take the weighing paper and remove the tare weight. Weigh 0.2 g KCl powder, 0.2 g KH2PO4 powder, 8 g NaCl particles, and 2.08 g Na2HPO4∙2H2O powder and place it in 2 L. In a glass beaker, add ultrapure water to make the volume to 1 L and place it on the shaker and vortex to dissolve, and after the solution is fully dissolved and mixed, pipette into a 1 L glass bottle, use concentrated hydrochloric acid solution and sodium hydroxide particles to adjust the pH of the PBS solution. The value reaches 7.4. After the preparation is completed, the bottle cap is fully wrapped in tin foil and loosened slightly until it does not fall off, place it in an autoclave at 121°C for 30 minutes, tighten the cap and place it in a refrigerator at 49°C, and store it at low temperature.

Preparation of MTT reagent: use a precision balance to weigh 0.5 g of MTT powder, dissolve it in 100 mL, pH = 7.4 phosphate buffer to prepare a 5 mg/mLMTT solution, filter it with a 0.22 um filter membrane in a sterile ultraclean table to remove the bacteria in the solution, divide it into a 10 mL centrifuge tube, wrap it with tin foil, and store it in a 49°C refrigerator in the dark to ensure sterility and convenient use.

#### 3.1.2. Breast Cancer Cell Proliferation and Culture

When the cell proliferation reaches 80%–90% of the bottom area of the culture flask, it is resuspended for passage, cryopreserved, and resuscitated according to experimental needs. The 4T1 was cultured by conventional methods. Take out the 4T1 breast cancer cell line, put it in a 37–40°C water bath, continuously vibrate the cryopreservation tube, add 5 ml RPM-1640 complete medium, and centrifuge at 100 pm for 5 minutes. Complete medium RPMI-1640 was added, transferred to a culture flask, and cultured in a CO_2_ incubator at 37°C. Observe every day, pay attention to pollution, changes in the color of the culture medium, cell attachment, and proliferation, etc, and change the medium with 0.25% pancreatin digestion every 3–4 days. Usually, every other day, it is necessary to observe changes in cell proliferation, including cell morphology. It is necessary to record the movement of cells and take photos in time, which can understand the changes in cell proliferation more comprehensively and in detail. Observe cells in a good proliferation state through a microscope, with high transparency and strong refraction intensity, and the microstructure of a part of the cells will be clearly visible. The growth of the cells is not good, the refraction of the cells is weak, and the gap between the cells becomes larger. Next, add 0.25% trypsin to the logarithmic phase attached cell culture flask used in the experiment to digest for 1 to 2 minutes. Place the culture flask in the microscope to shrink the cytoplasm and increase the intercellular space. The cells were pipetted in the suspension and centrifuged at 100 RPM for 5 minutes.

RETRACTED

### 3.2. Ultrasonic Irradiation Device

The ultrasonic irradiation in this experiment was produced by the CZ906A ultrasonic cavitation therapy instrument (Sichuan Mianyang Sonic Electronics Co., Ltd.). According to the in vitro cell experiment of the previous experiment, the parameters were set as follows: frequency 1 MHz, duty cycle 50%, action time 1 min, power 1 W/cm^2^; in vivo animal experiment setting parameters are frequency 1 MHz, duty cycle 50%, action time 1 min, and power 2 W/cm^2^. The in vitro experiment operations are all carried out in a sterile cell ultraclean table. The ultrasound probe is fixed in a water tank filled with sterilized double-distilled water. A 6-well plate is placed on the platform of the probe. The center of the probe is aligned with the target hole to ensure a small part of the bottom of the culture plate. Immerse under the liquid surface to prevent air bubbles between the ultrasound probe and the bottom of the orifice plate from affecting the experimental results; in vivo experiments, the probe is aimed at the tumor area of the nude mouse, and an appropriate amount of ultrasound coupling agent is used to conduct the sound velocity between the probe and the skin of the tumor site of the nude mouse conduction to avoid air bubbles.

With different ultrasonic irradiation intensities (0.5 W/cm^2^, 0.75 W/cm^2^, 1 W/cm^2^, and 1.25 W/cm^2^) and different irradiation times (10 s, 30 s, 45 s, and 60 s), the logarithmic growth phase of MCF-7, without any treatment, and the cells were cultured normally. Observe the influence of different ultrasound parameters on cell growth activity, and find out the most suitable combination of ultrasound intensity and irradiation time. Each group is equipped with four reholes to eliminate the influence of accidental experiment.

RETRACTED

### 3.3. Establishment and Grouping of 4T1 Breast Cancer Xenograft Model in BALB/c Mice

#### 3.3.1. Establishment of Breast Cancer Xenograft Model

4T1 breast cancer cells in the logarithmic proliferation phase were collected. After 0.25% was digested with pancreatin, it was washed twice with PBS to adjust the concentration to 1 × 10^7^/mL. A 0.1 mL tumor grows subcutaneously on the edge of the mouse chest, thereby establishing a breast cancer model of BALB/c mice. After 6–15 days, the tumor grows rapidly, and the growth volume of the tumor is measured with a vernier caliper. When the length of the tumor is 2.5 × 2.5, the modeling is successful.

#### 3.3.2. Grouping of Mice

Tumor-forming mice were randomly divided into the following four groups, each with 6: A. control group, B. safflower yellow group, C. ultrasound irradiation group, D. ultrasound irradiation combined with safflower yellow group. All tumor-forming mice were required to take dexamethasone every day for three days before receiving safflower yellow intervention treatment to prevent allergic reactions and fluid retention. The intervention measures are shown in Table 1.

### 3.4. Record the Quality Changes of Mice and the Measurement of Transplanted Tumor Volume and Tumor Inhibition Rate

From the second day of inoculation to the end of the experiment, the body weight of the mice successfully inoculated with 4T1 cells was measured every day; from the 5th day, tumors in each group were calculated body volume and tumor inhibition rate (TIR) of each group.

### 3.5. Organization and Testing

#### 3.5.1. Organize Materials

After 5 interventions, the mice were dislocated and sacrificed. The breast tumor tissue was completely removed and washed with normal saline, and the tumor tissue was cut into tissue specimens about 1 cm × 0.5 cm in size. Put a part of the tumor tissue in a refrigerator at 4°C, fix it with 4% formaldehyde for 24 hours, and put it in 5%, 10%, and 15% sucrose for dehydration. Finally, the tissue was placed in a refrigerator at −80°C for immunofluorescence calibration. The remaining tumor tissues were put directly into the refrigerator at −80°C for Western blot analysis.

#### 3.5.2. Determination of Protein Content

 
*Prepare Protein Standards*. Take the aliquoted 10uL BSA protein standard solution with a concentration of 5 mg/mL, add 90 *μ*l PBS diluent to it to obtain a protein standard with a concentration of 0.5 mg/mL; take the previously lysed protein solution with a pipette 5 *μ*L plus 45*μ*PBS diluent diluted 10 times to prevent the protein content from being too high; the OD value exceeds the protein standard curve, and the determination result is inaccurate; BCA working solution is configured. According to the needs of the experiment, calculate the amount of BCA working solution needed, and mix the Cu^2+^ reagent and BCA reagent in a 50 : 1 ratio according to the instructions until the flocs disappear for subsequent experiments.
 
*Protein Concentration Determination*. According to the instructions, add protein standards to the 96-well plate, add the volume of 0, 1, 2, 4, 8, 12, 16, and 20 uL, and then add 5 *μ*L and 10 *μ*u of diluted protein to ensure that the dilution of 20 is measured in the future. The protein OD value is 40 times and 40 times, and each concentration is set with 3 auxiliary holes to reduce the error. After adding the protein, the volume of the tested Luo solution is made up to 20 *μ*L with PBS diluent. This process tries to avoid bubbles. Then, add 200 uL of the previously configured BCA working solution to all the protein-containing well plates, place it in a 37°C constant temperature oven to avoid light for 15–20 min, then use a microplate reader to measure the OD value at 562 nm, draw according to the obtained OD value protein standard curve, and calculate the resulting protein concentration.
 
*Protein Denaturation and Preservation*. Set the protein concentration after denaturation to 4 ug/uL, add the calculated volume of protein, buffer, and lysate, wrap the centrifuge tube with a sealing strip, and place it in 100°C boiling water for 10 minutes to ensure that the protein is denatured and transferred to a 4C centrifuge. Centrifuge at 1000 rpm for 5 min, then blow out the protein samples uniformly, dispense them into 200 *μ*L centrifuge tubes according to the volume of 40 *μ*L per tube, and store the labeled protein information in a 20°C refrigerator.

RETRACTED

### 3.6. Detection of Cell Cycle

According to the above experimental method, the cells with good growth conditions are routinely made into a cell suspension. After the cell count, the cell suspension is diluted, and the cell suspension is inoculated in a six-well plate at a cell density of 25 × 104 cells/mL. Place the six-well plate on a sterile ultraclean table at 37°C for 24 hours and let it stand overnight, and wait for the cells to adhere to the wall stably; after the cells are stable, remove the six-well plate, place it on the sterile ultraclean table, take an appropriate amount of HSYB mother liquor to prepare 100 *μ*g/mL HSYB working solution, aspirate the old medium, add HSYB working solution to the final concentration of 0, 10, 20, 30 *μ*g/mL, keep the volume of the medium in the well plate at 3 mL, and shake the six-well plate to place the drug culture in a 37°C sterile incubator; 24 hours after the administration, the cells were routinely digested and collected. When the digestion was terminated, the cell supernatant was used to terminate the digestion. In addition to the concentration gradient group, there was another control group. After 30 minutes of 37°C water bath, add 400 *μ*L of PI staining solution to mix, incubate in a 49°C refrigerator in dark for 30 minutes, and then load the sample for measurement.

### 3.7. Statistical

The statistical processing of the data used SPSS21.0 software. Variance is used for comparison between groups, repeated measurement variance is used for comparison at different time points within a group, and the X test is used for comparison of count data. The rank total test is used for normally distributed count data. The statistical validity of this study was set as *P* < 0.05, and the statistical reasoning level of 5% was evaluated as meaningful.

## 4. Results and Discussion

### 4.1. Ultrasound Irradiation and Safflower Yellow on Cells

The survival rate of cells decreases with the increase of the ultrasonic intensity and the extension of the action time. When the intensity of ultrasonic irradiation is less than 1 W/cm^2^ and the time is less than 45 seconds, the cells are safe. When the ultrasonic intensity is 0.75 W/cm^2^, 45 seconds irradiation or 1 W/cm^2^ irradiation, 30 seconds of irradiation, the survival rate of breast cancer cells is only 10%, which is the most suitable ultrasonic parameter. The cell survival rate under different ultrasonic irradiation gas intensities is shown in Table 2.

Ultrasound (US) imaging is cost-effective and provides high resolution and excellent contrast for delineating soft tissue targets other than those that are obscured by the lungs or skull. Therefore, it is increasingly used in the verification of RT settings to measure movement between small joints. Ultrasound examination of breast cancer is shown in Figure 2.

First, the cytotoxicity of different concentrations of safflor yellow to tumor cells (10–100 *μ*g/mL) was tested. According to data analysis, it was found that the inhibition rate of 60 *μ*g/mL after the administration concentration did not change significantly, so the concentration gradient of the administration was adjusted as follows: 5, 10, 15, 20, 25, 30, 35, 40 *μ*g/mL, and we can see from Figure 2 that after 24 hours of administration, it was found that compared with the control group, the safflor yellow treated cells were tumor cells. The survival rate of serotonin is obviously inhibited, and the degree of inhibition exists in a concentration-dependent manner with the administration concentration. At the same time, the IC50 is determined to be between 20.4 *μ*g/mL, so we determined the experimental concentration to be 10, 20, and 30 *μ*g/mL. In this way, the next in vitro experiment was carried out. Inhibition rates of the cells treated with safflower yellow pigment were 14.6 ± 2.3%, 29.1 ± 2.9%, 33.7 ± 2.1%, 43.9 ± 3.8%, 61.2 ± 3.1%, 78.4 ± 2.9%, 84.4 ± 2.8%, and 87.4 ± 3.2%. The data prove that safflower yellow pigment can significantly inhibit the proliferation of tumor cells, and the inhibitory effect exists in a concentration-dependent manner. The inhibitory effect of different concentrations of safflor yellow on tumors is shown in Figure 3.

RETRACTED

### 4.2. 4T1 Breast Cancer Xenograft Model in BALB/c Mice

The tumor formation rate of mice was 100%, and the tumor formation time was 6 days after inoculation with 4T1 breast cancer cells. When the mice were first planted with breast cancer cell lines, the body weight of the mice did not change significantly, but with the passage of time, the body weight of the mice changed slightly. And the mice began to lose weight. The body weight changes of mice are shown in Figure 4.

The level of CD4^+^CD25 Foxp3^+^Treg in breast cancer of BALB/c mice on the 4th day after irradiation treatment decreased significantly (*P* < 0.05). The level of CD4^+^CD25 Foxp3^+^Treg in breast cancer of BALB/c mice on the 8th and 12th day after radiotherapy was lower than that before ultrasound treatment, and the trend was not obvious. Compared with the change of tumor body CD4^+^CD25 Foxp3^+^Treg grade, the change in the lymph node is not obvious. This may be related to the degree and size of lymph node metastasis and measurement errors. The electronic scan of breast cancer cells is shown in Figure 5.

The growth of transplanted tumors in each group of mice is shown in Figure 6. Among them, the growth rate of the control group was the fastest. The growth rates of transplanted tumors in the safflower yellow group, low-frequency ultrasound group, and the combination are slower, and some of the transplanted tumors in the treatment group tended to gradually stop growing.

The tumor growth of mice in each group is shown in Table 3. The tumor inhibition rate of the ultrasound irradiation and combination group was higher than that of the safflower yellow group, and the tumor inhibition rate of the combination treatment group was higher than that of the ultrasound irradiation group. It shows that both ultrasound irradiation and safflower yellow pigment can inhibit the growth of tumors. Ultrasound irradiation has a stronger tumor growth inhibitory effect than safflower yellow pigment, and the combination of the two has the best effect on inhibiting tumor growth.

RETRACTED

CD34-labeled MVD is Pearson related to Notch1, MMP-9, and VEGF protein expression, and the correlation coefficients *r* are 0.856, 0.723, and 0.809, respectively (*P* < 0.05), indicating that the CD34-labeled microvessel density in tumor tissue is correlated with Notch1, MMP-9, and VEGF protein expression are positively correlated, and this correlation is statistically significant. The CD34-labeled tumor tissue is shown in Figure 7.

## 5. Conclusion

This study mainly explores the antitumor proliferation and related mechanisms of ultrasound irradiation combined with safflower yellow. The breast cancer cell line 4T1 derived from BALB/c mice was selected. When the cell proliferation reached 80%–90% of the bottom area of the culture flask, it was resuspended, passaged, frozen, and resuscitated according to experimental needs. The 4T1 breast cancer cell line was cultured by conventional methods. 4T1 breast cancer cells in the logarithmic proliferation phase were collected. After 0.25% was digested with pancreatin, it was washed twice with PBS to adjust the concentration to 1 × 10^7^/mL. A 0.1 mL tumor cell suspension was subcutaneously inoculated on the edge of the mouse chest, thereby establishing a breast cancer model of BALB/c mice. After 6–15 days, the tumor grows rapidly, and the growth volume of the tumor is measured with a vernier caliper. When the length of the tumor is 2.5 × 2.5, the modeling is successful. From the second day of inoculation, body weight of the mice successfully inoculated with 4T1 cells was measured every day; from the 5th day, the tumors in each group were calculated body volume and tumor inhibition rate (TIR) of each group. Ultrasound irradiation combined with safflower yellow pigment can effectively inhibit tumor proliferation. The occurrence of tumors is an interaction of multiple factors. While using traditional Chinese medicine treatment, it should be actively combined with chemotherapy, radiotherapy, and targeted drugs. The combination of therapy and surgery can better improve the curative effect, prolong the life cycle of patients, and improve the quality of life of patients healed.

## Figures and Tables

**Figure 1:** Ultrasonic irradiation equipment (http://alturl.com/dut3r).

**Figure 2:** Ultrasound examination of breast cancer (http://alturl.com/g4og7).

RETRACTED

**Figure 3:** The inhibitory effect of different concentrations of safflor yellow on tumors.

**Figure 4:** Changes in mouse body weight.

**Figure 5:** Electronic scan of breast cancer cells (http://alturl.com/jyt67).

**Figure 6:** The growth of transplanted tumors in each group of mice.

**Figure 7:** CD34-labeled tumor tissue (http://alturl.com/e6vmz).

**Table 1:** Interventions.

Groups	Intervention method
Group A	Inject normal saline (0.3 ml) via tail vein
Group B	Docetaxel (7.5 mg/kg) via tail vein injection every other day
Group C	Low-frequency ultrasound irradiation for 5 min(0.75w/cm^2^, 1.0 MHz, duty cycle 2.0%)
Group D	B + C

**Table 2:** Cell survival rate under different ultrasonic irradiation gas intensities.

Ultrasonic intensity (W/cm^2^)	Ultrasound action time (s) and cell survival rate (%)			
	10	30	45	60
0.5	96.40	94.76	94.12	93.33
0.75	94.06	93.20	90.63	85.87
1.0	92.19	90.75	86.87	82.69
1.25	85.18	75.27	63.36	55.49

**Table 3:** Tumor growth of mice in each group.

Group	Tumor (mm^3^)	Tumor inhibition rate (%)
Control group	2192 ± 341	0
Safflower yellow group	1603 ± 336	28.5 ± 12.4
Low-frequency ultrasound group	1211 ± 289	45.6 ± 10.1
Drug + ultrasound group	975 ± 106	55.6 ± 4.3
*F* value	3.631	8.933
*P* value	0.031	0.001

## Data Availability

No data were used to support this study.
